The article "Kinetic Gait Changes after Robotic Exoskeleton Training in Adolescents and Young Adults with Acquired Brain Injury" was published in 2020. Journal: Appl Bionics Biomech.

# Kinetic Gait Changes after Robotic Exoskeleton Training in Adolescents and Young Adults with Acquired Brain Injury

**DOI:** 10.1155/2020/8845772

**Published:** 2020-10-27

**Authors:** Kiran K. Karunakaran, Naphtaly Ehrenberg, JenFu Cheng, Katherine Bentley, Karen J. Nolan

**Affiliations:** ^1^Center for Mobility and Rehabilitation Engineering Research, Kessler Foundation, West Orange, New Jersey 07052, USA; ^2^Physical Medicine and Rehabilitation, Rutgers New Jersey Medical School, Newark, New Jersey 07103, USA; ^3^Research Department, Children's Specialized Hospital, New Brunswick, New Jersey 08901, USA

## Abstract

**Background:**

Acquired brain injury (ABI) is one of the leading causes of motor deficits in children and adults and often results in motor control and balance impairments. Motor deficits include abnormal loading and unloading, increased double support time, decreased walking speed, control, and coordination. These deficits lead to diminished functional ambulation and reduced quality of life. Robotic exoskeletons (RE) for motor rehabilitation can provide the user with consistent, symmetrical, goal-directed repetition of movement, as well as balance and stability.

**Purpose:**

The goal of this preliminary prospective before and after study is to evaluate the therapeutic effect of RE training on the loading/unloading and spatial-temporal characteristics in adolescents and young adults with chronic ABI.

**Method:**

Seven participants diagnosed with ABI between the ages of 14 and 27 years participated in the study. All participants received twelve 45 minute sessions of RE gait training. The bilateral loading (linearity of loading and rate of loading), speed, step length, swing time, stance time, and total time were collected using Zeno™ walkway (ProtoKinetics, Havertown, PA, USA) before and after RE training.

**Results:**

Results from the study showed improved step length, speed, and an overall progression towards healthy bilateral loading, with linearity of loading showing a significant therapeutic effect (*p* < 0.05).

**Conclusion:**

These preliminary results suggest that high dose, repetitive, consistent gait training using RE has the potential to induce recovery of function in adolescents and young adults diagnosed with ABI.

## 1. Introduction

Acquired brain injury (ABI) is a leading cause of hemiparesis resulting in gait and balance deficits in adolescents and young adults [1–3]. These deficits result in abnormal loading and unloading, increased double support time, and decreased walking speed, control, and coordination, leading to impairment in functional ambulation and associated activities of daily living [2–5]. Recovery involves rehabilitation through high dose physical therapy [6]. It is based on the theory that the human brain is capable of self-reorganization, or plasticity, through continuous, consistent, repeated practice aimed at restoring function and independence [7–9]. Conventional therapy alone may not be able to provide enough consistent mass practice and repetition to facilitate the neuroplasticity needed for a functional recovery [10]. Consequently, after motor rehabilitation individuals with ABI can experience variable recovery with residual gait deviations. As a result of these residual motor and balance deficits, individuals diagnosed with ABI may develop compensatory mechanisms such as abnormal or asymmetrical loading and unloading characteristics and prolonged weight transfer, in order to achieve ambulation [4, 11].

Ground reaction force (GRF) parameters, e.g., peak values, linearity, and rates of loading/unloading, symmetry coefficients, and force integrals, are used for assessment of pathological gait and evaluation of therapeutic efficacy [12–14]. The analysis of vertical forces during gait provides information on weight bearing and balance, and these force or pressure patterns in the paretic leg are known to be correlated with walking speed and motor recovery in stroke patients [15, 16]. Therefore, improvements in vertical pressure profiles might demonstrate improvement in gait and overall functional ambulation.

In a healthy gait cycle, the loading response is bilaterally symmetrical [17]. It has three distinct phases, starting with a peak force during the initial loading phase, followed by a midstance phase where there is a decrease in loading, and ending with another peak force during the terminal unloading phase [17]. Thus, the loading response resembles a bimodal M shape [17]. The transfer of weight during the initial loading phase allows for the efficient transfer of momentum from one leg to the other and the uninterrupted use of the kinetic energy that is created by swing limb activity [18]. The rate of loading determines the speed of gait [15]. Research has shown that smooth linear loading helps conserve momentum and shifts the body's weight to the next phase of the gait cycle while maintaining speed [14, 17, 19]. If weight transfer is delayed or loading is nonlinear, it will result in a loss of energy and hence less efficient gait, leading to decreased speed and necessitating the use of other compensatory gait mechanisms. Limb loading is often inefficient in individuals with ABI because the affected limb has a difficult time accepting weight, resulting in a nonlinear loading and decreased momentum. Consequently, a targeted goal during gait rehabilitation in ABI is to improve loading profiles in order to facilitate healthier movement patterns.

Lower extremity robotic exoskeletons (REs) are currently being used in rehabilitation to restore gait functionality. REs have the potential to provide the user with high dose, consistent, symmetrical bilateral loading [9, 20–26] profiles during gait. It can provide an increased number of steps (increased dosing) in a consistent and controlled training environment, which is ideal for inducing neuroplasticity [20, 27]. This is essential for chronic ABI patients who need high dose, consistent therapy to induce cortical reorganization for functional recovery. This study utilized an RE to provide intensive gait training to adolescents and young adults diagnosed with an ABI, with the goal of evaluating the efficacy of high repetition robotic training on loading/unloading profiles. The objective of this preliminary prospective study was to evaluate the therapeutic effect of RE on their loading/unloading characteristics. This paper also provides details of the RE gait training environment for reference, to help understand the therapeutic effects.

## 2. Materials and Methods

This is a preliminary prospective before and after study which is to evaluate the therapeutic effect of RE training on the loading/unloading and spatial-temporal characteristics in adolescents and young adults with chronic ABI.

### 2.1. Participants

Twelve participants with ABI were recruited for this study. Kinetic and temporal-spatial data for baseline and follow-up visits were only available from nine participants. Further, two participants were excluded from the analysis as they were diagnosed with bilateral deficits. Therefore, seven participants diagnosed with ABI and hemiparesis and a single healthy control (HC) were included for this analysis (Table 1). The inclusion criteria for ABI participants in this investigation included (1) diagnosed with an acquired brain injury (anoxic, stroke, or TBI); (2) between the ages of 13 and 28; (3) able to walk with or without an assistive device; (4) no additional orthopedic, neuromuscular, or severe neurological pathologies (unrelated to their ABI) that would interfere with their ability to walk; (5) able to stand upright for 30 minutes with assistance; and (6) able to physically fit into the RE (weight ≤ 100 kg, height ≤ 1.88 m, hip width 0.36 m-0.46 m). The inclusion criteria for the HC were no orthopedic, neuromuscular, or severe neurological pathologies that would interfere with gait and balance. All procedures performed in this investigation were approved by the Human Subjects Institutional Review Board at Kessler Foundation, and informed consent was obtained prior to study participation.

### 2.2. Robotic Exoskeleton Gait Training

Robotic gait training in bilateral assistance mode was administered as an outpatient rehabilitation gait intervention at the Kessler Foundation using a commercially available robotic exoskeleton (Figure 1, EksoGT, Ekso Bionics, Inc., Richmond, CA, USA) for 45 minutes per day for 12 days over a period of 4 weeks. A licensed physical therapist administered all RE gait training sessions and adjusted the assistance provided by the robot to the individual participant's therapy progression. A member of the study team was present at all times during the RE gait training sessions to assist the physical therapist and ensure participant safety. The healthy control participant was not given RE training as part of the investigation.

The RE provided overground gait rehabilitation under the guidance of a licensed physical therapist. The RE's upper section is attached to the user's upper body, with a backpack style shoulder harness and torso brace and also houses the battery pack, while the lower sections are affixed to the legs with upper thigh straps, shin guards, and secure foot bindings. The RE has two active degrees of freedom at the hip and the knee, respectively, and a passively sprung ankle joint with adjustable stiffness in the sagittal plane. The RE provides assistive torques to the hip and knee joints to perform the predefined gait trajectory and provides variable assistance as required by the participants bilaterally. The actuated range of motion at the hip is -20° to 135°, and the actuated range for the knee is 0° to 120° [28]. All steps were initiated by the participant. In order to trigger a step, the subject performed a lateral weight shift to a predetermined distance from midline to initiate advancement of the back (preswing) leg.

### 2.3. Data Collection Procedures

The participants with ABI participated in two data collection sessions (baseline and follow-up after 12 sessions of outpatient RE training), and data was collected while walking with (training environment) and without the RE. The participants with ABI did not utilize any orthotic devices or dorsiflexion wrap during data collection. The reference HC participated in one data collection session, and data was collected while walking without the RE.

During each data collection session, temporal, spatial, and loading data was collected using a Zeno™ walkway (ProtoKinetics, Havertown, PA, USA) at 120 Hz. The participant performed up to 6 walking trials (approximately six 10 meter walks) at a self-selected pace per condition (with and without RE) and wore shoes for all walking assessments. Participants were allowed to rest or take breaks at any time during testing to minimize the effects of fatigue. A member of the study team was present with the participants at all times during the walking trials.

During the baseline and follow-up gait assessments in the RE, torque was provided bilaterally as needed at the hip and knee to complete the gait.

### 2.4. Data Analysis

PKMAS (ProtoKinetics Havertown, PA, USA) and MATLAB (MathWorks, Natick, MA, USA) were used for data analysis. The data were preprocessed using the PKMAS software, and temporal, spatial, and normalized pressure data were exported. Custom MATLAB algorithms were used to analyze the gait trajectories for each session with and without the RE. The exported data were further divided into gait cycles, with a gait cycle being defined as the period from ground contact of one foot to the subsequent ground contact of the same foot. Data for up to 15 gait cycles per condition and per session were available for each subject and were used for data analysis. Selected outcome measures and statistical analyses are presented in Table 2.

## 3. Results

### 3.1. Total Vertical Pressure (TVP)

Figure 2 shows the average TVP of all participants with ABI at baseline and at follow-up for both the affected and the unaffected sides with and without RE and one reference HC. The reference HC's TVP profile demonstrated linear loading and unloading, a symmetrical loading pattern during stance bilaterally, and a minimal deviation from the mean across gait cycles. For participants with ABI walking without RE at baseline, the TVP demonstrated a perturbation during loading for the IDS phase (Figure 2-P1and Figure 3-P3) and increased loading on the unaffected side. At follow-up, the perturbation during loading for IDS decreased (Figure 2-P2 and Figure 3-P3), and there was increased loading on the affected limb during midstance. There was increased variation in the TVP on the affected side compared to the unaffected side for individuals with ABI, demonstrated by the standard deviations.

In the RE training environment, the TVP profile showed linear loading during IDS, but did not show the distinctive peaks as observed in the HC's data (Figure 2-VP1 and Figure 2-VP3) in both the affected and unaffected sides at both baseline and follow-up. Furthermore, a bilaterally symmetrical loading profile was observed in the RE training environment and for the HC as compared to without RE. The deviation from the mean across gait cycles for participants with ABI was smaller in the RE training environment compared to without the RE at both baseline and follow-up.

### 3.2. Rate of Linear Loading (Slope of Initial Loading)

There was an increase in the average slope from baseline to follow-up while walking without the RE (Table 3). A paired sample *t*-test for average slope did not show a significant therapeutic effect between baseline and follow-up, though the effect size (*p* = 0.136, Cohen's *d* effect size was 0.59) was high (Table 3). The average slope was higher in the training environment (with the RE) both at baseline and at follow-up compared to without the RE. The RE training environment was similar to HC (Table 3).

### 3.3. Linearity of Loading (Goodness of Fit)

There was an increase in average *R*^2^ from baseline to follow-up while walking without the RE (Table 3). The Wilcoxson signed rank test for *R*^2^ showed a significant therapeutic effect between baseline and follow-up, and the effect size (*p* = 0.018, Cohen's *d* effect size was 0.6334) was high. The *R*^2^ of loading was higher in the training environment (with the RE) at baseline and about the same at follow-up compared to without the RE. The RE training environment was similar to the HC (Table 3).

### 3.4. Step Length

Step length without the RE showed an increase in both the unaffected and affected sides at follow-up compared to baseline in subjects 2,3,5,6, and 7, while it showed a decrease in subject 1 and no change on the unaffected side and an increase on the affected side in subject 4 (Figures 2(a) and 2(b)). A paired sample *t*-test did not show a significant therapeutic effect between baseline and follow-up, though the effect size (*p* = .075, Cohen's *d* effect size was 0.81) was high. The average step length was lower in the training environment (with the RE) compared to without the RE at baseline and follow-up. The average step length of the HC data was higher than ABI without RE.

### 3.5. Walking Speed

Walking speed without the RE increased from baseline to follow-up for subjects 2,4,5,6, and 7, while subject 1 decreased their speed, and subject 3 showed no change (Figure 2(c)). A paired sample *t*-test did not show a significant therapeutic effect between baseline and follow-up, though the effect size (*p* = 0.083, Cohen's *d* effect size was 0.80) was high. The average walking speed was lower in the training environment (with the RE) compared to without the RE at baseline and follow-up. The average speed of the HC data was higher than ABI without RE.

### 3.6. Temporal Characteristics

Average total time, stance time, and total double support time decreased from baseline to follow-up (Table 4), but did not show a significant therapeutic effect (*p*_totaltime_ = 0.612, *p*_stance time_ = 0.398, *p*_total double support time_ = 0.237). The average total time, stance time, and total double support time were higher in the training environment (with the RE) compared to without the RE at baseline and at follow-up. Average total time, stance time, and total double support time of the HC data were lower than ABI without RE.

Swing time did not change (*p* = 0.866) from baseline to follow-up (Table 4). The average swing time was higher in the training environment (with the RE) compared to without the RE at baseline and follow-up. Average swing time of the HC data was lower than ABI without RE.

## 4. Discussion

Moderate to severe ABIs may result in gait and balance deficits such as reduced speed, step length, and abnormal loading and unloading characteristics during walking. Current research is focused on reducing these deficits with the use of REs and understanding the therapeutic effects of REs in the chronic stages of recovery. Recovery may be gradual during the chronic stages and may take place over the course of several years. In this study, the efficacy of RE usage for 12 sessions on the recovery of gait in adolescents and young adults with chronic ABI was investigated using kinetic and temporal-spatial outcomes, such as loading, unloading, speed, step length, and gait cycle timing. Following the use of the RE, an increase in linearity of loading during IDS with an associated increase in speed, step length, and decrease in stance phase time was observed.

During a healthy gait cycle, the loading/unloading response is bilaterally symmetrical, as is observed in Figure 2. It has three distinct phases. The role of the first phase is the weight acceptance which includes initial contact (heel strike) and the initial loading response. This is the initial double support phase of the gait cycle and starts with heel strike and continues until the contralateral foot is in swing [17]. The second phase supports the upper body on a single limb, and it is comprised of midstance and terminal stance (single support phase). The third phase includes preswing and the terminal unloading phase [17]. Distinct peaks and a valley are observed in the loading profile during these phases, with a peak force (Figure 2-VP1) at the end of the initial loading, followed by a midstance and terminal phase where there is a decrease in loading (Figure 2-VP2) and ending with another peak force (Figure 2-VP3) before terminal unloading [29]. In addition, bilaterally symmetrical loading profiles are present. These attributes are observed in the reference HC gait. In contrast, the individuals with ABI had a perturbation during initial loading (Figure 2-P1, Figure 3-P3) on the affected side during baseline, which indicates a nonlinear initial loading response. Linear loading directly contributes to the momentum during gait [30]. Therefore, any nonlinearity would result in decreased momentum and slower load transfer during gait, leading to a disruption in forward progression. ABI patients with hemiplegia often present with reduced hip flexion, dorsiflexion, and plantarflexion during the initial loading phase due to muscle paresis [11, 31]. This results in the tibia not rolling forward over the calcanium, which is observed as non-linearity, to complete the transfer of the body weight from the contralateral limb [11]. In this study, linearity of loading was quantified using goodness of fit, which showed that the individuals with ABI had a statistically significant improvement in the linearity of their loading responses at follow-up compared to baseline (Figure 2-P2, Figure 3-P4, and Table 3). This may indicate that the participants have healthier foot strike, and initial loading response with improved momentum, at follow-up compared to baseline. The slope of the initial loading response showed an increase at follow-up compared to baseline (Table 3). Although the difference was not significant, it had a high Cohen's *d* effect size at follow-up compared to baseline, indicating that the participants had improved their rate of loading, once again, demonstrating preserved forward momentum. Thus, at follow-up, TVP showed an increase in smooth linearity and rate of loading similar to healthy individuals [17]. Research has shown that improved linearity and slope during loading result in improved gait pattern, resulting in improved functional ambulation and quality of life [14]. Also, improvements in initial loading may reduce breaking forces [32], leading to a more efficient gait. Though the participant's overall loading profiles showed improvements from baseline to follow-up, they still preferentially loaded their unaffected side.

The loading profile with the RE showed a smooth linear loading (Figure 3), but without any distinctive peaks. A passive ankle in the RE (which provides a midfoot or flat foot landing) or lower speed may have resulted in the absence of two distinctive peaks. Changes in walking speed may improve this profile and need to be investigated further. In addition, a bilaterally symmetrical profile with lower variability was observed at both baseline and follow-up while walking with the RE compared to walking without the RE, indicating that the RE provides a consistent training environment throughout therapy. Thus, the improvements in the smoothness and linearity of loading could be attributed to the RE training. Our results are in accordance with previous research which showed that with the use of overground RE, there was an increased bilateral limb loading symmetry that closely resembled able-bodied gait [33, 34].

In addition, after 12 sessions of RE gait training, there was a slight increase in the step length and an increase in walking speed (Figure 4(a)). There was no change in swing time and a decrease in stance time. These results suggest that the increased step length (Figure 4(a)) and improved TVP profile may have contributed to the increased walking speed (Figure 2(a)). They are significant since most of the participants in this study were walking below the community ambulation speed (1 m/s) [35]. An increase in speed could improve their community ambulation and by extension, their activities of daily life. Previous research on overground gait training with RE has shown the ability of RE to improve balance and functional ambulation in patients with ABI [36, 37]. Overground REs require active participation, where patients initiate each step and are responsible for maintaining trunk and balance [21, 37]. Active participation in combination with RE's ability to provide quality gait and increased dose training promotes improved brain plasticity and connectivity remodulation, as compared to conventional gait training [21, 38, 39].

This is one of the first studies to show the feasibility of using RE for gait training in adolescents and young adults with ABI. The results from this preliminary study show a therapeutic effect of RE on the loading/unloading characteristics and a consequent impact on functional ambulation. Although these results are promising, the limitations of this investigation are the limited sample size, number of training sessions, and absence of control group. The data from this study indicates some promising results for therapeutic effects of an RE device for ABI gait rehabilitation that should continue to be explored with a larger sample.

## 5. Conclusion

The results from this investigation suggest that improvement in functional and neuromechanical outcomes after 4 weeks of RE gait training can be achieved in adolescents and young adults with chronic ABI. This study suggests that there could be potential long-term effects of improved loading and unloading, increased step length, and increased speed due to RE gait training. While the current results are promising, future studies with a larger sample would be required to further understand the efficacy of the RE in adolescents and young adults to confirm any training effect conclusively.

## Figures and Tables

**Figure 1:** Robotic gait training with a participant with ABI administered by a trained physical therapist.

**Figure 2:** Mean ± standard deviation of the TVP of the affected and unaffected leg of individuals with ABI during walking with and without an RE at baseline and follow-up and one reference HC. Data is normalized to 100% of the stance phase.

**Figure 3:** Mean ± standard deviation of the initial loading phase of the right and left leg of subjects with ABI while walking with and without the RE at baseline and at follow-up and a reference HC. The dotted lines are the best fit lines for the loading profile.

**Figure 4:** Mean ± standard error of the step length with and without the RE on the (a) affected side, (b) unaffected side, and (c) walking speed.

**Table 1:** Subject demographics.

Subject	Condition	Affected side	Gender	Age	Height (m)	Weight (Kg)	Years since injury
1	TBI	Left	Male	23	1.83	90.00	1
2	Stroke	Left	Female	23	1.60	54.00	.9
3	Anoxic	Left	Female	17	1.63	54.00	2
4	Stroke	Left	Male	16	1.83	67.50	.5
5	TBI	Left	Male	22	1.78	63.50	3
6	TBI	Left	Female	27	1.63	62.60	5
7	TBI	Right	Male	14	1.65	49.44	0.5

Mean ± SD				20.29 ± 4.68	1.71 ± 0.10	63.01 ± 13.51	1.84 ± 1.66

1	HC	n/a	Male	26	1.57	77.11	n/a

**Table 2:** Outcome measures.

Outcome measure	Description	Statistical analysis
Total vertical pressure (TVP)	TVP during the stance phase of each gait cycle was computed, and an average TVP for all gait cycles was calculated for both the legs without and with RE that was computed for each subject and for the HC. The TVP was normalized to 100% of stance in each condition for comparison. The stance phase was further divided into initial double support (IDS) and terminal double support (TDS) phases based on heel strike and toe off. The IDS pressure was computed as the pressure between ipsilateral heel strikes to contralateral toe off. The TDS pressure was computed as the pressure between contralateral heel strikes to ipsilateral toe off. Mean and standard deviation TVP for all participants with ABI was computed.	
Linearity of loading (goodness of fit)	A best fit line was computed for the average IDS loading phase for each session for each subject. A goodness of the fit was computed to assess the error between the fitted line and the average loading during IDS for each subject in each session. The goodness of fit was used to assess the smooth linearity of loading. *R*-square (*R*^2^) was computed to assess the square of the correlation between average loading during IDS and the best fit line. A higher *R*^2^ value signifies a closer fit to the best fit line or increased linearity.	Kolmogorov- Smirnov *Z* test (*p* < 0.05) of normality showed that the data were not normal. Wilcoxson signed rank test was used to determine the therapeutic effect (baseline to follow-up without RE) on goodness of fit.
Rate of linear loading (slope of initial loading)	The slope of the average IDS loading phase was computed for each subject. Slope indicates the rate of linear loading. Increased slope in the IDS phase indicates an increased moment during the first rocker.	Kolmogorov- Smirnov *Z* test (*p* > 0.05) of normality showed that the data were normal. A paired sample *t*-test was performed to determine the therapeutic effect (baseline to follow-up without RE) on the slope of initial loading.
Walking speed	The average walking speed was computed for each subject as the linear distance with respect to time to complete a gait cycle.	Kolmogorov- Smirnov *Z* test (*p* > .05) of normality showed that the data were normal. A paired sample *t*-test was performed to determine the therapeutic effect (baseline to follow-up without RE) on walking speed.
Step length	The average step length for each gait cycle was computed as the forward linear displacement between foot contact of the ipsilateral leg to foot contact of the contralateral leg during each gait cycle. Average step length was computed for each subject.	Kolmogorov- Smirnov *Z* test (*p* > .05) of normality showed that the data were normal. A paired sample *t*-test was performed to determine the therapeutic effect (baseline to follow-up without RE) on step length.
Temporal measures	Total time was computed as the time between foot contact of one leg to the subsequent foot contact of the same leg. The average total time was computed for each gait cycle. Further, average swing time for each subject during each condition was computed as the time between the foot off the floor of one leg to foot contact of the same leg during the gait cycle. Average stance time for each subject during each condition was computed as the time between the foot contact of one leg to toe off the same leg during the gait cycle.	Kolmogorov- Smirnov *Z* test (*p* < .05) of normality showed that the data were not normal. Wilcoxson signed rank test was used to the therapeutic effect (baseline to follow-up without RE) on total time, swing time, and stance time.

**Table 3:** Mean ± standard error of initial double support (IDS) loading characteristics on the affected side of all participants with ABI and IDS loading characteristics on the left side of one HC.

Metric	Baseline-without RE	Follow-up-without RE	Baseline-with RE	Follow-up-with RE	HC
Slope	2.33 ± 0.28	2.60 ± 0.36	3.44 ± 0.29	3.43 ± 0.24	3.46
Goodness of fit	0.889 ± 0.05	0.934 ± 0.04	0.927 ± 0.02	0.923 ± 0.02	0.99

**Table 4:** Mean ± standard error of temporal characteristics.

	Metric	Baseline-without RE	Follow-up-without RE	Baseline-with RE	Follow-up-with RE	HC
Affected	Total time	2.18 ± 0.69	1.98 ± 0.50	3.78 ± 0.17	3.35 ± 0.09	1.24
	Stance time	1.66 ± 0.62	1.46 ± 0.45	3.12 ± 0.15	2.69 ± 0.10	0.80
	Swing time	0.52 ± 0.07	0.52 ± 0.06	0.66 ± 0.05	0.66 ± 0.06	0.44
	Total double support	1.25 ± 0.62	1.05 ± .045	2.40 ± 0.17	2.04 ± 0.10	0.36

Unaffected	Total time	2.15 ± 0.66	1.95 ± 0.48	3.77 ± 0.16	3.33 ± 0.10	1.27
	Stance time	1.74 ± 0.66	1.55 ± 0.47	3.05 ± 0.17	2.69 ± 0.10	0.85
	Swing time	0.41 ± 0.04	0.40 ± 0.04	0.72 ± 0.11	0.64 ± 0.02	0.43
	Total double support	0.73 ± 0.49	0.44 ± 0.21	1.19 ± 0.10	1.01 ± 0.05	0.23

## Data Availability

The data is currently unavailable due to Kessler Foundation IRB restrictions.
